RETRACTED

# Prevention of Dexmedetomidine on Postoperative Delirium and Early Postoperative Cognitive Dysfunction in Elderly Patients Undergoing Thoracoscopic Lobectomy

**DOI:** 10.1155/2022/5263021

**Published:** 2022-10-14

**Authors:** Jing Zhao, Wei-Bo Wang, Hui Ding, Hua-Jun Fu, Yan-An Jiang

**Affiliations:** ^1^Department of Anesthesiology, Shaanxi Provincial People's Hospital, Xi'an 710068, Shaanxi, China; ^2^Department of Anesthesiology, Shaanxi Provincial Pucheng Country Hospital, Weinan 715500, Shaanxi, China

## Abstract

**Objective:**

To investigate the effect of dexmedetomidine on postoperative cognitive function and delirium in elderly patients undergoing thoracoscopic lobectomy.

**Methods:**

109 elderly patients (age is more than 65 years) who underwent thoracoscopic lobectomy in our hospital from June 2020 to Feb 2022 were randomly divided into the dexmedetomidine (DEX) group (*n* = 54) and the control group (*n* = 55). The patients in the experimental group were given dexmedetomidine by intravenous pump, intravenous pump 0.5 *μ*g/kg within 10 minutes, and maintained the speed of 0.5 *μ*g/(kg. h) to 30 min before the operation was ended. The control group was given the same amount of normal saline. Delirium assessment-severity (CAM-S) assessment and Mini-Cog were used to assess the severity levels of POD and POCD 24 h before, 6 hours after, one day after the operation, three days after the operation, and 1 week after the operation. Serum TNF-*αα* and NSE levels were assessed by using enzyme-linked immunosorbent assay. NRS pain marks were assessed in the DEX group at postanesthesia care unit (PACU) and 24 postoperation. Surgical pierhysmographic index (SPI) evaluation was performed at five time points.

**Results:**

The Mini-Cog scores in the DEX group were markedly enhanced compared with those in the saline group 6 and 24 hours after the operation. The SPI values in the DEX group were markedly reduced within 2 min after intubation and at surgical sutures. Moreover, the CAM scores in the DEX group were markedly reduced 24 hours after the operation. Tumor necrosis factor-*α* (TNF-*α*) and neuron-specific enolase (NSE) levels were significantly decreased in the DEX group at T1∼T3.

**Conclusion:**

The use of dexmedetomidine in the thoracoscopic lobectomy in elderly patients could reduce the occurrence and severity of postoperative cognitive dysfunction and delirium.

## 1. Introduction

Postoperative delirium (POD) and postoperative cognitive dysfunction (POCD) are the common manifestations of acute brain dysfunction after general anesthesia and surgical operation [1, 2]. Particularly for elderly patients, POD and POCD are more likely to occur after an operation [3]. Notably, it has been indicated recently that the incidence of POD and POCD in elderly patients after thoracic surgery were 32% and 19%, respectively [4, 5].

RETRACTED

Lung cancer is one of the common malignant tumors, and its morbidity and mortality rates are still on the rise [6]. Lobectomy is the primary treatment for early lung cancer [7]. Lobectomy aims to remove the diseased lobes and clean up the lymph nodes to inhibit the spread of cancer cells and prolong the survival time of patients [8]. Intrathoracic operation is tightly associated with severe aches, and unacceptable postsurgical pain administration might hinder convalescence and increase the hazards of POD and POCD [9]. Notably, it has been exposed recently that efficient postsurgical analgesia might diminish the danger of POD following cardiac operation [10]. Several reports have exhibited that a more excellent postsurgical pain score correlates with the augmented POD hazard [11].

Dexmedetomidine (DEX) is an efficient and intensely optional *α*2-adrenergic receptor agonist and functions as a polyfunctional medication in healing numerous human sicknesses [12]. As reported previously, DEX effectively treats neural disorders by diminishing central nervous sympathetic efflux and offering calm and analgesia [13]. In addition, DEX usage might ameliorate behavioral turbulences, such as an attack, anxiety, and cognitive dysfunction [14]. Moreover, several reports have suggested DEX has anesthetic, minor tranquilizer, and antidelirium properties without agitation [15]. These characteristics make it a proper selection for sedation in the clinic.

Primary research with mice models has indicated that DEX protects the nervous system and ameliorates rates of cognitive function after the operation [16, 17]. Several clinical research studies have suggested the favorable impact of DEX in ameliorating postsurgical cognitive diminishing, whereas others could not observe similar results [18]. However, it remains uncertain whether the application of DEX could ameliorate POD and POCD in elderly patients undergoing thoracoscopic lobectomy. To obtain the newest evidence, our study widely assesses whether DEX could improve postoperative delirium and early postoperative cognitive dysfunction in elderly patients undergoing thoracoscopic lobectomy.

## 2. Materials and Methods

### 2.1. Patients

Qualified elderly patients (>65 years) with long cancer after thoracoscopic lobectomy from June 2020 to Feb 2022 in Shaanxi Provincial People's Hospital were enrolled in the current study. Inclusion criteria are as follows: ① age 65∼80; ② United States American Society of Anesthesiologists, ASA grade I ∼ II; ③ Preoperative selfrating Depression Scale (SDS) score >53; ④ the patients were well tolerated to dexamethasone and planned to undergo thoracic surgery under general anesthesia; ⑤ patients were clinically diagnosed as lung cancer; and ⑥ all patients signed informed consent.

RETRACTED

Exclusion criteria are as follows: ① patients were diagnosed with preoperative cognitive impairment; ② severe liver and kidney dysfunction; ③ previous cardiovascular and cerebrovascular diseases or central nervous system diseases; ④ patients were unable to communicate generally due to difficulties in expression; ⑤ unable to complete thoracoscopic lobectomy; ⑥ pulmonary ventilation dysfunction or pleural adhesion; and ⑦ thoracoscopic surgery failed and thoracotomy was selected.

### 2.2. Anesthesia Management

The patients in the experimental group were given dexmedetomidine (Yangtze River Pharmaceutical Group Co Ltd) by intravenous pump, intravenous pump 0.5 *μ*g/kg within 10 minutes, and maintained the speed of 0.5 *μ*g/(kg. h) to 30 min before the operation was ended. The control group was given the same amount of normal saline. Intravenous-inhalation general anesthesia was induced by propofol (Xi'an Libang Pharmaceutical Co Ltd) (2.0∼2.5 mg/kg), sufentanil (Yichang Renfu Pharmaceutical Co Ltd, 0.3 *μ*g/kg), and rocuronium (Zhejiang Xianju Pharmaceutical Co Ltd, 0.6 mg/kg). After tracheal intubation, sevoflurane (Shanghai Hengrui Pharmaceutical Co Ltd, 2% ∼ 3%) and remifentanil 0.2 *μ*g/(Yichang Renfu Pharmaceutical Co Ltd, kg·min) and propofol 4∼5 mg/(kg·h) are pumped intravenously to maintain anesthesia. The bispectral index (BIS) was maintained during anesthesia at 45∼60. Pressure-controlled ventilation was used for mechanical ventilation during one-lung ventilation. Control the peak airway pressure <25 cm H_2_O.

### 2.3. POD Assessment

POD was evaluated by a validated confusion assessment method (CAM) [19]. This scale had high sensitivity (94% ∼ 100%) and specificity (90% ∼ 95%). CAM evaluation included acute changes or fluctuations in the state of consciousness, attention defect, incoherent thinking, and change of consciousness. Delirium assessment-severity (CAM-S) assessment was used to assess the severity levels of POD, with a score of 0∼7. Scoring criteria are as follows: 0 for normal, 1 score for mild delirium, 2 scores for moderate delirium, and 3-7 for severe delirium.

### 2.4. POCD Assessment

POD was evaluated by the Mini-Cog 24 h before the operation, 6 hours after the operation, 1 day after the operation, 3 days after the operation, and 1 week after the operation. Mini-Cog is a cognitive assessment, which comprises a memorial assignment implicating the remembrance of three words and the assessment of a clock drawing mission [20]. The higher the score is, the better the cognitive function.

RETRACTED

### 2.5. Serum TNF-*α* and NSE Assessment

Peripheral blood was collected after anesthesia and before operation (T0), induction (T1), on the opening vessel bypass time (T2), 2 h after the end of the operation (T3), and then centrifuged at 3500 r/pm for 15 minutes. The separated serum is stored in the refrigerator at −20°C. Serum TNF-*α* and NSE levels were assessed by using enzyme-linked immunosorbent assay (Shanghai Qiaoyu Biological Co Ltd).

### 2.6. Statistical Analysis

Data were evaluated by SPSS 20.0 and GraphPad Prism software. Quantifiable statistics were represented as mean ± standard deviation (SD). Comparison between groups was assessed by Student's *t*-test or Mann–Whitney *U* test. Repetitive measurement of variance testing with Bonferroni correction was employed to evaluate the concentrations of TNF-*α* and NSE at specific times. The difference was statistically significant (*P* < 0.05).

## 3. Results

### 3.1. Sufferers' Characteristics

A total of 102 elderly sufferers were recruited for this research. Three sufferers were excluded owing to changing to thoracotomy. Ultimately, 54 sufferers were admitted to the DEX group and 55 to the S (saline) group. No differences in age, sex, ASA condition, weight, height, smoking history, extubating timing, and BMI were observed between patients in the DEX and saline groups (Table 1). Furthermore, anesthesia and artificial pneumothorax timing did not differ between the DEX group and saline group.

### 3.2. Surgical Pierhysmographic Index Evaluation

The surgical pierhysmographic index (SPI) evaluation exhibited that the SPI values before the operation, at endotracheal intubation, and during surgical incision did not differ between the DEX group and saline group (Figure 1). Moreover, the SPI values in the DEX group were markedly reduced within 2 minutes after intubation and at surgical sutures compared with the saline group (*P* < 0.05, Figure 1).

### 3.3. NRS Pain Index

NRS pain marks in the saline group were markedly enhanced compared with those in the DEX group at PACU (*P* < 0.05, Figure 2). Moreover, there existed no notable differences in pain marks between the DEX group and saline group 24 hours postoperation, suggesting that DEX could effectively reduce NRS pain index in PACU.

### 3.4. Neurocognitive Function Measurement

The Mini-Cog scores in the DEX group were markedly enhanced compared with those in the saline group 6 hours after the operation (*P* < 0.05, Table 2). The Mini-Cog scores in the DEX group were remarkably increased compared with those in the saline group 24 hours after the operation (*P* < 0.05; Table 2). However, the Mini-Cog scores did not differ between the DEX and saline groups at other inspection times (Table 2).

RETRACTED

Moreover, the CAM scores in the DEX group were markedly reduced compared with those in the saline group 24 hours after the operation (*P* < 0.05, Table 3). The DEX and saline groups detected no differences in the other CAM parameters (Table 3).

### 3.5. Occurrence of Adverse Events

The incidence of bradycardia in the DEX group was markedly higher than that in the saline group (*P* < 0.05), and there was no significant difference in the incidence of hypotension, hypertension, and allergy between the DEX group and S group (Table 4).

### 3.6. The Incidence and Severity of POD and POCD

The incidence of POD in the DEX and saline groups was 11.1% and 27.3%, respectively. The incidence of POD in the DEX group was lower than in the S group (*P* < 0.05). The incidence of POCD in the DEX and saline groups was 16.7% and 30.9%, respectively. The incidence of POCD in the DEX group was lower than in the S group (*P* < 0.05). There was no significant difference in the incidence of POD severity and days of POCD per individual between the DEX group and S group (Table 5).

### 3.7. Serum TNF-*α* and NSE Levels

No differences in the serum TNF-*α* and NSE levels were observed between the DEX and saline groups before operation (Figure 3). Compared with the saline group, the TNF-*α* and NSE levels were significantly decreased in the DEX group at T1∼T3 (all *P* < 0.05).

## 4. Discussion

In recent years, many studies have paid attention to postoperative delirium and postoperative cognitive dysfunction after the operation [21]. Elderly patients undergoing major thoracic surgery have a higher probability of postoperative delirium and postoperative cognitive dysfunction [22]. As a clinical treatment for lung cancer and other serious lung diseases, lobectomy could effectively remove the focus and save the patient's life. Lobectomy has the disadvantages of considerable trauma, long operation time, and surgical solid stress response, which might seriously affect the patient's respiratory function and bring many complications [23]. POD and POCD are common complications after lobectomy [24]. Therefore, active prevention and treatment of POD and POCD have always been a concern.

As a new imidazole derivative, dexmedetomidine has high selectivity for *α*2 receptor and could effectively activate *α*2 receptor [25]. Pharmacological studies have suggested that its biological potency is better than clonidine. Compared with traditional sedative drugs such as propofol and midazolam, dexmedetomidine mainly acts on the locus coeruleus nucleus instead of the cerebral cortex, effectively avoiding the critical points of sedation and anxiety [26]. Therefore, the risk of postoperative anxiety is significantly reduced by dexmedetomidine. In the current study, we observed that DEX could decrease the incidence and severity of POCD and POD in elderly patients undergoing thoracoscopic lobectomy, which validated its capability to guard against delirium and cognitive dysfunction following the operation.

RETRACTED

The elders would remain increase smoothly in the next few years. With enlarged age, people undergo more repeatedly from illnesses and suffer frequently encountered disease [27]. Furthermore, the occurrence of cognitive destruction in the elders is not to be undervalued. Delirium is a common complication after surgical operation in elderly patients. It is the acute onset accompanied by disturbance of consciousness and change of mental state [28]. In the present study, we used a validated confusion assessment method (CAM) to evaluate the effect of dexmedetomidine on postoperative POD in elderly patients undergoing thoracoscopic lobectomy. We found that DEX could reduce the incidence and severity of POD in elderly patients undergoing thoracoscopic lobectomy. Mini-Cog is one of the most used criteria for evaluating the cognitive function of patients undergoing thoracic surgery. As a standard clinical assessment approach to POCD, the Mini-Cog score is commonly applied in evaluating cognitive function. In the present study, we observed that Mini-Cog scores were higher in the DEX group than those in the saline group at 24 h preoperatively; 6 h, 24 h, and 72 h postoperatively; and 1 week postoperatively. Continued postoperative transfusion with DEX could improve the Mini-Cog score during a small postoperative stage, suggesting that DEX could reduce the incidence and severity of POCD in elderly patients undergoing thoracoscopic lobectomy.

At present, the mechanism of perioperative neurocognitive impairment is unknown. Previous studies have shown that the inflammatory response resulting from perioperative surgical trauma and other factors is one of the critical causes of POD and POCD [29]. This study found that TNF-*α* and NSE levels in the DEX group at T0, T1, T2, and T3 were notably lower than those in the saline group. These findings indicated that intravenous dexmedetomidine infusion before anesthesia induction might reduce the inflammatory and stress response in patients undergoing thoracoscopic lobectomy.

In brief, intravenous dexmedetomidine infusion before anesthesia induction could reduce the incidence and severity of POD and POCD in patients undergoing thoracoscopic lobectomy. These findings of the current study indicated that dexmedetomidine might prevent postoperative POD and POCD in elderly patients undergoing thoracoscopic lobectomy. However, further studies are still needed to warrant the current conclusion.

RETRACTED

## Figures and Tables

**Figure 1:** SPI values before the operation, at endotracheal intubation, and during surgical incision in the DEX group and saline group.

**Figure 2:** NRS pain marks at PACU and 24 hours after operation in the DEX group and saline group.

**Figure 3:** Serum TNF-*α* and NSE levels in the DEX group and saline group.

**Table 1:** Sufferers' baseline characteristics.

Parameter	DEX group (*n* = 54)	S group (*n* = 55)	*P*
Age, year	63.01 ± 3.04	64.59 ± 4.02	0.261
Sex (no., %)			0.102
Female	30 (55.56%)	32 (58.18%)	
Male	24 (44.44%)	23 (48.82%)	
BMI (kg/m^2^)	26.01 ± 2.05	26.00 ± 2.33	0.559
ASA I/II (no., %)	6 (11.11%)	8 (14.55%)	0.291
Weight, kg	65.02 ± 5.33	64.00 ± 4.27	0.311
Height, cm	167.01 ± 5.60	168.00 ± 4.96	0.201
Smoking history	10.02 ± 3.05	9.97 ± 4.19	0.708
Anesthesia timing, min	203.56 ± 34.90	209.56 ± 40.03	0.089
Artificial pneumothorax timing, min	81.02 ± 12.05	88.09 ± 13.40	0.402
Extubating timing, min	18.09 ± 5.04	18.01 ± 4.98	0.907

Data are described as mean ± SD or amount (percentage).

**Table 2:** Comparison of Mini-Cog score between the DEX group and saline group.

	DEX group (*n* = 54)	S group (*n* = 55)	*P*
24 hours before the operation	26.84 ± 0.87	27.98 ± 0.73	0.102
6 hours after the operation	23.90 ± 1.03	21.42 ± 2.93	0.002
24 hours after the operation	26.31 ± 1.32	25.08 ± 1.09	0.019
72 hours after the operation	27.45 ± 0.82	27.69 ± 0.93	0.338
1 week after the operation	28.01 ± 1.53	28.34 ± 0.87	0.056

Data are described as mean ± SD.

**Table 3:** Comparison of CAM score between the DEX group and saline group.

	DEX group (*n* = 54)	S group (*n* = 55)	*P*
24 hours before the operation	16.24 ± 1.29	16.68 ± 1.08	0.703
6 hours after the operation	20.95 ± 1.03	21.01 ± 1.53	0.398
24 hours after the operation	19.31 ± 1.46	19.78 ± 1.25	0.012
72 hours after the operation	17.45 ± 1.32	17.89 ± 1.13	0.508
1 week after the operation	16.24 ± 1.43	16.35 ± 1.27	0.256

Data are described as mean ± SD.

**Table 4:** Comparison of incidence of adverse events between the DEX group and saline group.

	DEX group (*n* = 54)	S group (*n* = 55)	*P*
Bradycardia/[cases (%)]	8 (14.8)	13 (23.6)	0.011
Hypotension/[cases (%)]	7 (12.9)	15 (27.3)	0.098
Hypertension/[cases (%)]	4 (7.4)	1 (1.8)	0.078
Allergy	2 (3.7)	1 (1.8)	0.508

Data are described as the amount (percentage).

**Table 5:** Comparison of POD and POCD incidence and severity between the two groups.

	DEX group (*n* = 54)	S group (*n* = 55)	*P*
POD incidence, *N* (%)	6 (11.1)	15 (27.3)	0.004
POCD incidence, *N* (%)	9 (16.7)	17 (30.9)	0.008
POD severity (score)	2.4 ± 1.1	2.2 ± 1.0	0.084
Days of POCD per individual, *N* (%)	0.6 ± 0.7	0.4 ± 0.5	0.208

Data are described as mean ± SD or amount (percentage).

RETRACTED

## Data Availability

The labeled datasets used to support the findings of this study are available from the corresponding author upon request.
